# Ultrasonic Image Restoration Algorithm for Prevention of Nervous Disorders during the Recovery Period of Patients Receiving Sevoflurane Anesthesia

This article has been retracted.

**DOI:** 10.1155/2021/6124346

**Published:** 2021-10-01

**Authors:** Gong Chen, Jinquan Yang, Qin Chen, Damin Liu

**Affiliations:** Department of Anesthesia Operation, Maternal and Child Health Care Hospital of Hunan, Changsha,410008, Hunan, China

## Abstract

In this article, dexmedetomidine (Dex) was used to prevent neurological disorders in patients anesthetized with sevoflurane and the effect was analyzed using ultrasound images based on the restoration algorithm of the linear system model. Children injected with Dex were in the experimental group, while children injected with normal saline were in the control group. The mean arterial pressure (MAP), arterial oxygen saturation (SpO_2_), heart rate (HR), Pediatric anesthesia agitation scale (PAED) score, Face, Legs, Activity, Cry, Consolability (FLACC) score, and adverse drug event (ADE) in the two groups were compared before the injection (T1), at 5 min (T2), 10 min (T3), and 20 min (T4) after the injection, and when the patient came to himself (T5). It was found that in contrast with the control group, the MAP in the experimental group at T2, T3, and T4 periods was lower, while it was higher at T5 period and its HR at T2, T3, T4, and T5 periods was higher (*P* *<* 0.05); the PAED and FLACC scores were lower (*P* *<* 0.05), and the incidence of ADE (10.53%) was lower than that in the control group (31.58%) (*P* *<* 0.05). However, SpO_2_ at different periods showed no obvious differences between the two groups (*P* *>* 0.05). In conclusion, the restoration algorithm-based ultrasound images had high quality, and they demonstrated good application value in evaluating the effect of Dex to prevent neurological disorders in patients anesthetized by sevoflurane.

## 1. Introduction

Ultrasonic imaging is an acoustic technology based on ultrasonic pulse reflection, which uses the ultrasonic beam to generate reflected signals at the interface of tissues and then obtains the images of internal organs [1]. Although ultrasonic imaging is real-time, safe, and nondestructive, it has low resolution and low contrast compared with CT and MRI. The main reason is that the tissue reflectivity and point spread function (PSF) convolve and accumulate noise [2]. Therefore, ultrasonic image restoration is necessary to enhance the definition of images. In recent years, many scholars have dedicated in research on ultrasonic image restoration technology and achieved remarkable results. In the process of ultrasonic image restoration, the size and shape of the PSF influence the outcome of the restoration. Dalitz et al. [3] studied the application of deconvolution in ultrasonic image restoration based on PSF. It was found that the PSF can be calculated using a simple closed analytic term based on the far-field approximation instead of a numerical value.

Inhalation anesthesia has been used clinically since a hundred years. Inhalation anesthesia is usually used for the induction and maintenance of anesthesia in pediatric operations. Sevoflurane is an anesthetic drug with relatively stable induction. Because of its fast induction of anesthesia, no irritating smell, and low blood distribution coefficient, it is more suitable for pediatric anesthesia. At present, sevoflurane is widely used clinically [4, 5]. Related studies have shown that the incidence of sevoflurane emergency agitation is as high as 20%–80%. Emergency agitation during the recovery period may cause bleeding, tracheal tube displacement, prolapse, and other conditions. Therefore, it is of great importance [6, 7]. Clinical studies have proved that propofol, amine tablets, etc. cannot obviously reduce the emergency agitation of children [8, 9]. Dex, as a highly selective *α*_2_ receptor agonist, is widely used in sedation, analgesia, and antianxiety. It can act on *α*_2_ receptors to inhibit the release of norepinephrine, thereby achieving sedation, analgesia, and antianxiety [10]. Relevant studies have shown that 1 *μ*g/kg Dex can reduce the incidence of emergency agitation in children and maintain good hemodynamics of children in operation [11].

To sum up, to obtain high-quality ultrasound images and better assist doctors, it is necessary to improve the original ultrasound images through ultrasonic image restoration technology. In the study, the linear model of ultrasound images and the working principle of the Field II ultrasound simulation platform were adopted for analysis. Then, the Field II method was used to estimate the PSF. Finally, the ultrasound image was restored by the deconvolution restoration method. Sevoflurane inhibits the respiratory function of children, while Dex drugs not only can reduce the pain and stress response of children but also have no significant inhibition on the respiratory function of children. Therefore, based on the ultrasonic image restoration, the effect of Dex was investigated on preventing sevoflurane emergency agitation in children.

## 2. Materials and Methods

### 2.1. Selection of Research Samples

In this study, 76 children undergoing tonsillectomy were selected as the research subjects, who were admitted to the hospital from February 2018 to January 2019. They were between 3 and 10 years old and rolled into a control group (38 cases) and an experimental group (38 cases) in random. In the control group, there are 25 males and 13 females, with an average age of (6.13 ± 2.78) years. In the experimental group, there were 23 males and 15 females, with an average age of (6.35 ± 2.89) years. The study has been approved by the medical ethics committee of the hospital, and the patients and their family members were informed and signed consent forms.

Inclusion criteria were as follows: (i) patients older than 2 years; (ii) patients classified as I and II by ASA; (iii) patients who have not received surgical treatment; (iv) patients younger than 11 years; (v) patients undergoing normal examination with consciousness.

Exclusion criteria were as follows: (i) patients with mental illness; (ii) patients with liver and kidney dysfunction; (iii) patients allergic to sedative drugs; (iv) patients with incomplete clinical data; (v) patients who withdrew from the experiment due to their own reasons.

### 2.2. Ultrasound Image Restoration Algorithm

The PSF and the tissue reflectivity convolve and accumulate the noise. The restoration process of ultrasound images can be described with a linear system model. The ultrasound image restoration can be expressed as follows:

(1) $$\begin{array}{c} G\left(x,y\right)=K\left(x,y\right)*P\left(x,y\right)+U\left(x,y\right), \end{array}$$

where *x* and *y* represent the horizontal and vertical coordinates, respectively, *∗* represents a discrete two-dimensional linear convolution operator, *G* (*x*, *y*) represents the received ultrasonic radio-frequency (RF) data, *K* (*x*, *y*) is a two-dimensional point-diffusion function, *P* (*x*, *y*) is the tissue-reflectivity image, and *U* (*x*, *y*) represents additive noise and is assumed to be white noise.  Figure 1 shows the classical linear model of ultrasonic imaging. The restoration process of ultrasonic images was the process from *G* (*x*, *y*) to *P* (*x*, *y*).

PSF estimation is the key step in the ultrasound image restoration. In the study, the Field II method was adopted to study the two-dimensional PSF, which was based on the Field II ultrasonic simulation platform. It was assumed that the PSF is constant in the lateral direction and variable in the axial direction. Therefore, the received RF echo data can be segmented axially. The PSF corresponding to each segment can be estimated by the Field II method. Then, each segment accepted deconvolution restoration, and all segments after the deconvolution and restoration were put together to form the final image. The unconstrained inverse filtering deconvolution restoration method is adopted.

After Fourier transform was performed on both sides of equation (1), the following equation is obtained:

(2) $$\begin{array}{c} G\left(a,b\right)=K\left(a,b\right)P\left(a,b\right)+U\left(a,b\right), \end{array}$$

where *G*(*a*, *b*), *P*(*a*, *b*), *U*(*a*, *b*), and *K*(*a*, *b*) are the Fourier transform of the observed image *G(x*, *y)*, the tissue-reflectivity image *P*(*x*, *y*), noise *U*(*x*, *y*), and point-diffusion function *K*(*x*, *y*). According to equation (2), the equation of tissue-reflectivity image in the frequency domain is obtained:

(3) $$\begin{array}{c} P\left(a,b\right)=\frac{G\left(a,b\right)}{K\left(a,b\right)}-\frac{U\left(a,b\right)}{K\left(a,b\right)}. \end{array}$$

When there is no noise, equation (3) can be expressed as follows:

(4) $$\begin{array}{c} P\left(a,b\right)=G\left(a,b\right)\frac{1}{K\left(a,b\right)}. \end{array}$$

In this way, the estimate of the tissue-reflectivity image *P*(*x*, *y*) can be obtained by performing Fourier Transform on *P*(*a*, *b*). The1/*K*(*a*, *b*) in equation (4) can be considered as a filter, and 1/*K*(*a*, *b*) is just the reverse of the imaging system *K*(*a*, *b*). Therefore, the process is called the inverse filtering restoration method. The following equation is obtained by performing inverse Fourier transform on equation (4):

(5) $$\begin{array}{c} P\left(x,y\right)=P^{-1}\left[P\left(a,b\right)\right]=P^{-1}\left[G\left(a,b\right)\frac{1}{K\left(a,b\right)}\right]. \end{array}$$

### 2.3. Comparison of Methods to Estimate PSF

Since the estimation of the PSF is a key step of ultrasound image restoration, in the study, the complex cepstrum method [12] and the generalized homomorphic filtering method [13] were introduced for comparison. The three fragments of 5, 10, and 20 were selected for comparison. In this study, the Field II estimation method was used as a reference. The errors generated by PSF were estimated using the generalized homomorphic filtering method and the complex cepstrum method. The mean square error (MSE) was introduced for measurement, and the equation is as follows.

(6) $$\begin{array}{c} MSE=\frac{1}{m{\left\|T_{r}\right\|}_{F}^{2}}\sum_{i=1}^{m}{\left\|T_{r}-T_{i}\right\|}_{F}^{2}. \end{array}$$

In equation (6), *T*_*r*_ represents the real PSF, *T*_*i*_ is the estimated value of PSF *i*, *m* represents the total times of estimation, and *F* represents the norm of the Frobenius matrix.

The MSE produced by PSF estimated by the generalized homomorphic filtering method and complex cepstrum method can be calculated by equation (6).

### 2.4. Methods of Anesthesia

All patients underwent fasting for 4 hours and were forbidden to drink for 2 hours before the operation, and no drugs were taken. Before the operation, the patients' intravenous trocar should be indwelled, and oxygen and aspiration devices, first aid drugs, and equipment should be prepared. In the operating room, the patients' routine blood pressure, blood oxygen, etc. were checked. Both groups of patients were treated with sevoflurane (Shanghai Hengrui Pharmaceutical Co., Ltd., China) according to the standard. After the patients lost consciousness, an intravenous channel was established for intravenous injection of 0.1 mg/kg of vecuronium (Jiangsu Enhua Pharmaceutical Co., Ltd., China) and 2 *μ*g/kg of fentanyl (Sinopharm Group Industry Co., Ltd., China). Then, tracheal intubation was performed, and an anesthesia machine (Drager Fabius, Germany) was employed to control the breathing mechanically. Patients in the experimental group were given 1 *μ*g/kg.h Dex (Jiangsu Hengrui Pharmaceutical Co., Ltd., China) by continuous intravenous pump injection, and patients in the control group were given the same amount of normal saline. After the operation, the sevoflurane inhalation and Dex pumping were stopped.

### 2.5. Observation Indicators

The MAP, SpO_2_, and HR in the two groups were detected with Philips VE24 (USA) before the injection (T1), at 5 min (T2), 10 min (T3), and 20 min (T4) after the injection, and when the patient came to himself (T5). After the drug was stopped, the children were sent to the resuscitation room and awakened 10 minutes later. The nursing staff used a single-blind method to evaluate the child's PAED and FLACC scores. The scoring criteria of PAED were as follows: no restlessness scored less than 5 points; mild restlessness scored 5–10 points; severe restlessness scored 10–15 points. FLACC is a scale used to assess the degree of pain in infants and children who cannot confirm the pain/quantify the degree of pain. Its takes account of expressions, leg movement, body position, crying, and comfort. The lowest score is 0, which means there is no pain. Mild pain scores 1–4 points, obvious pain scores 5–8 points, and severe pain scores 9–10 points. The occurrence of ADE and its incidence after surgery were recorded.

### 2.6. Statistical Methods

The data were processed by SPSS19.0, the mean ± standard deviation (‾*x* ± *s*) illustrated how to calculate the measurement data, and the count data were expressed as a percentage. MPA, SpO_2_, HR, and PAED scores during anesthesia between the two groups were compared by the paired *t*-test. Analysis of variance was adopted for comparison among groups. The difference was statistically significant with *P* *<* 0.05.

## 3. Results

### 3.1. Descriptive Statistics of Basic Data

Statistics on the basic conditions of the two groups of children, such as gender, age, weight, anesthesia time, and operation time, revealed that there was no obvious difference in the basic conditions (*P* *>* 0.05) (Table 1).

### 3.2. Comparison of Methods to Estimate PSF

As shown in Figure 2, the MSEs of segments 5, 10, and 20 estimated by the complex cepstrum method were 0.178, 0.301, and 0.437, respectively, while those estimated by the generalized homomorphic filtering method were 0.136, 0.154, and 0.141, respectively. The PSF estimated by the Field II method was taken as a reference, and the MSEs generated by the PSF of the generalized homomorphic filtering method and the complex cepstrum method were compared. The MSE generated by the PSF estimated by the generalized homomorphic filtering method was obviously lower than that estimated by the complex cepstrum method (*P* *<* 0.05), indicating the PSF obtained by the generalized homomorphic filtering method was closer to the PSF estimated by the Field II method than the PSF obtained by the complex cepstrum method.

Since the PSF estimated by the Field II method was closer to the real PSF, it was selected to estimate the PSF in this study. Then, unconstrained inverse filtering deconvolution was adopted to restore ultrasound images. As shown in Figure 3, the middle cerebral artery, the terminal segment of the internal carotid artery, the anterior cerebral artery, and the posterior cerebral artery on one cerebral hemisphere were clearly visible.

### 3.3. Comparison of MAP and HR

As shown in Figure 4, the MAP values of the control group at T1, T2, T3, T4, and T5 periods were 70.53 ± 9.32, 76.13 ± 8.67, 77.79 ± 8.53, 78.67 ± 8.47, and 79.91 ± 8.65 (mm/Hg), respectively; those in the experimental group were 71.03 ± 8.26, 73.23 ± 7.73, 72.53 ± 8.37, 74.20 ± 8.19, and 86.83 ± 9.87 (mm/Hg), respectively. There was no obvious difference in MAP of the two groups at T1 (*P* *>* 0.05), while in contrast with the control group, the MAP values of the experimental group at T2, T3, and T4 periods were obviously lower, but value at T5 period was obviously higher (*P* *<* 0.05).

∗ indicated that the difference was obvious in contrast with the control group (*P* < 0.05) (with the same meaning in Figures 5–8).

The HRs of the control group at T1, T2, T3, T4, and T5 periods were 103.23 ± 17.35, 95.33 ± 16.68, 93.65 ± 17.47, 92.16 ± 16.91, and 106.74 ± 17.18 (times/min); those of the experimental group were 102.35 ± 18.58, 100.23 ± 17.85, 101.54 ± 18.12, 99.69 ± 18.24, and 126.86 ± 17.93 (times/min), respectively. As shown in Figure 5, there was no obvious difference in HR between the two groups at T1 period (*P* *>* 0.05), while the HRs of the experimental group at T2, T3, T4, and T5 periods were obviously higher (*P* *<* 0.05).

### 3.4. Comparison of SpO_2_

As shown in Figure 9, the SpO_2_ rates of the control group at T1, T2, T3, T4, and T5 periods were 99.31 ± 0.62, 98.23 ± 0.69, 98.67 ± 0.59, 99.30 ± 0.71, and 98.89 ± 1.02 (%), respectively; those of the experimental group were 99.47 ± 0.45, 99.25 ± 0.37, 98.69 ± 0.51, 98.58 ± 1.16, and 99.57 ± 0.34 (%), respectively. As shown in Figure 9, there was no obvious difference in SpO_2_ between the two groups at T1, T2, T3, T4, and T5 periods (*P* *>* 0.05).

### 3.5. Comparison of PAED and FLACC

As shown in Figure 6, the PAED scores of the control group at T1, T2, T3, T4, and T5 periods were 12.73 ± 4.67, 8.74 ± 4.28, 7.31 ± 3.91, 5.68 ± 4.12, and 3.95 ± 4.29 (minutes), respectively; those of the experimental group were 13.16 ± 5.17, 5.02 ± 3.67, 4.56 ± 4.17, 3.98 ± 4.65, and 3.59 ± 4.36, respectively. The PAED scores of the two groups at T1 and T5 were not obviously different (*P* *>* 0.05); while the PAED scores of the experimental group at T2, T3, and T4 periods were obviously lower than those of the control group (*P* *<* 0.05).

As shown in Figure 7, the FLACC scores of the control group at T1, T2, T3, T4, and T5 periods were 5.74 ± 2.13, 4.98 ± 2.08, 4.11 ± 1.79, 3.78 ± 2.25, and 2.98 ± 1.85 (points), respectively; those of the experimental group were 5.81 ± 1.97, 3.92 ± 2.35, 3.06 ± 1.37, 2.51 ± 1.69, and 2.05 ± 1.49 (minutes), respectively. As shown in Figure 7, there was no obvious difference between the FLACC scores of the two groups at T1 period (*P* *>* 0.05); however, the FLACC scores of the experimental group at T2, T3, T4, and T5 periods were obviously lower (*P* *<* 0.05).

### 3.6. Comparison of the Incidence of ADE

As shown in Figure 8, in the control group, there were 8 cases with coughing and 4 cases with vomiting after surgery, with a total of 12 cases of ADE, and the incidence of ADE was 31.58%. In the experimental group, there were 3 cases with cough and 1 case with vomiting after operation. There were 4 cases of ADE, and the incidence of ADE was 10.53%. It was evident that the incidence of ADE in the experimental group was obviously lower than that in the control group (*P* *<* 0.05).

## 4. Discussion

At present, ultrasound imaging technology is widely used in medical diagnosis and detection and has become the most commonly used method [14]. However, ultrasound imaging has low resolution and low contrast. In the restoration of ultrasound images, PSF is required to evaluate the quality of the image. Using the Field II method to estimate PSF can get a more accurate PSF [15] to improve the clarity of the image. Sevoflurane is a new type of anesthesia-inducing drug. Because of its strong controllability and low liver and kidney toxicity, it is widely used in pediatric surgical anesthesia [16]. However, some studies have found that children are prone to agitation after sevoflurane anesthesia. Dex is a highly selective *α*_2_ receptor agonist. It is mainly used for compound anesthesia, ICU sedation, preoperative medication, imaging-assisted examination, postoperative agitation prevention, etc. [17]. The application of Dex in pediatric anesthesia has not yet been fully demonstrated and is still at the theory level.

In the study, the PSF was estimated by the Field II method and the ultrasound image was restored by the deconvolution restoration method. Then, the effect of Dex was investigated on preventing sevoflurane emergency agitation in children. It was found that the PSF estimated by the Field II method was closer to the real PSF. Furthermore, the PSF obtained by the generalized homomorphic filtering method was closer to the PSF estimated by the Field II method than the PSF obtained by the complex cepstrum method. It was aligned with the research results of Jemec et al. [18]. High-resolution ultrasound images were obtained using the deconvolution algorithm. The MAP, SpO_2_, HR, and PAED and FLACC scores of the two groups at different time periods were detected; there was no obvious difference in MAP between the two groups at T1 period (*P* *>* 0.05), while the MAP of the experimental group at T2, T3, and T4 periods was lower and that at T5 was higher (*P* *<* 0.05). The HRs of the experimental group were 102.35 ± 18.58, 100.23 ± 17.85, 101.54 ± 18.12, 99.69 ± 18.24, and 126.86 ± 17.93 (times/min), respectively, and were higher than those of the control group at T2, T3, T4, and T5 periods (*P* *<* 0.05). There was no obvious difference in SpO_2_ between the two groups at different time periods (*P* *>* 0.05). The PAED and FLACC scores of the experimental group were significantly lower than those of the control group at T2, T3, and T4 periods (*P* *<* 0.05). The incidence of ADE in the experimental group was significantly lower than that in the control group (*P* *<* 0.05). This was similar to the results of Di et al. [19], suggesting that Dex can reduce the incidence of emergency agitation and ADE in children. In addition, the hemodynamic indicators of two groups were analyzed at different time points, and the results showed that the patient can maintain a good hemodynamic level during the operation.

## 5. Conclusion

In the study, the linear model of ultrasound images and the working principle of the Field II ultrasound simulation platform were adopted for analysis. The ultrasound images were restored by the deconvolution restoration method to obtain the ones with higher quality. On the basis of ultrasound image restoration, the effect of Dex was investigated on preventing sevoflurane emergency agitation in children. It turned out that Dex can effectively reduce the incidence of emergency agitation and the adverse conditions after the operation. However, the sample size is small, which may cause deviations in the results. In the follow-up studies, the number of patients will be increased to further explore the effect of Dex on preventing sevoflurane emergency agitation in children. In summary, the results provide a theoretical basis for the study of ultrasound image restoration algorithms and Dex's prevention of neurological disorders in patients undergoing sevoflurane anesthesia [20].

## Figures and Tables

**Figure 1:** Linear model of ultrasound imaging.

**Figure 2:** Comparison of MSE estimated by the two methods. ^*∗*^The difference was obvious in contrast with the complex cepstrum method (*P* *<* 0.05).

**Figure 3:** A cerebrovascular ultrasound image. The figure is cerebral vascular color Doppler ultrasound of an 11-year-old girl.

**Figure 4:** Comparison of MAP.

**Figure 5:** Comparison of HR.

**Figure 6:** Comparison of PAED scores.

**Figure 7:** Comparison of FLACC.

**Figure 8:** Comparison of the incidence of ADE.

**Figure 9:** Comparison of SpO_2._.

**Table 1:** Differences in the basic conditions.

	Boys (people)	Average age (years)	Weight (kg)	Anesthesia time (min)	Operation time (min)
Control group	25	6.13 ± 2.78	23.35 ± 4.23	54.76 ± 6.13	45.69 ± 7.36
Experimental group	23	6.35 ± 2.89	24.13 ± 3.52	55.21 ± 7.39	46.37 ± 8.12

## Data Availability

The data used to support the findings of this study are available from the corresponding author upon request.
